This article has been retracted.

# The Study of Face Processing in Social Anxiety Disorder Based on Face-Specific N170 Component

**DOI:** 10.1155/2022/6003973

**Published:** 2022-01-07

**Authors:** Xuejing Bi, Min Guo, Jianqin Cao, Yanhua Hao

**Affiliations:** ^1^Department of Nursing, Harbin Medical University, Daqing 163319, China; ^2^Academy of Electronic Information and Electrical Engineering, Xiamen Institute of Technology, Xiamen 361021, China; ^3^School of Health Management, Harbin Medical University, Harbin 150081, China

## Abstract

Although previous studies showed that social anxiety disorder (SAD) exhibits the attentional bias for angry faces, few studies investigated effective face recognition combined with event-related potential (ERP) technique in SAD patients, especially the treatment effect. This study examines the differences in face processing in SAD patients before and after treatment and healthy control people (H-group). High-density EEG scans were registered in response to emotional schematic faces, particularly interested in the face processing N170 component. Analysis of N170 amplitude revealed a larger N170 for P-group-pre in response to inverted and upright stimuli than H-group in the right hemisphere. The result of the intragroup *t*-test showed that N170 was delayed for inverted relative to upright faces only in P-group-post and H-group but not in P-group-pre. Remarkably, the results of ANOVAs manifested that emotional expression cannot modulate N170 for SAD patients. Besides, the N170-based asymmetry index (AI) was introduced to analyze the left- and right-hemisphere dominance of N170 for three groups. It was found that, with the improvement of patients' treatment, the value of *AI*_*N*170−*base*  *d*_ presented a decreasing trend. These results together suggested that there was no inversion effect observed for patients with SAD. The change in the value of *AI*_*N*170−*base*  *d*_ can be used as potential electrophysiological markers for the diagnosis and treatment effects on patients with SAD.

## 1. Introduction

Social anxiety disorder (SAD) is an anxiety disorder accompanied by both unusual physical and mental symptoms, mainly characterized by intense fear when facing social interaction context or public places. Previous studies have indicated that patients with SAD are associated with deficits in social cognition, including several cognitive biases such as expectation bias, attention bias, memory bias, and response bias to faces, even for neutral faces [1, 2]. For example, patients with SAD exhibit a more robust amygdala activation in response to neutral faces than healthy control individuals [3], while affective context can modulate the processing of neutral faces for patients with SAD [4]. Magnetoencephalography (MEG) study suggested that patients with SAD show reduced N170 representing early fusiform gyrus activity compared to healthy controls [5]. In contrast, an EEG study showed blunted early discrimination on faces that have rejected or accepted them [6]. Given the abnormality of SAD patients in face processing, the early-stage neural responses of patients with SAD may be different compared with healthy individuals and may also change with treatment.

Face perception plays an indispensable role in both social life and interpersonal communication. Even normal newborn babies tend to pay attention to face-related stimuli [7]. Damaging the face-related neural mechanism involved in face recognition can seriously affect everyday life. At the same time, other studies have indicated that social anxiety disorders showed avoidant and escaped responses to faces with direct eye contact [8, 9]. Recent research showed that cognitive-behavioral therapy can reduce the early visual processing of faces for patients with social anxiety disorder [10]. Although considerable effort has been made to study the neural processing of face-related information in mental disorders, including prosopagnosia, autism spectrum disorders (ASD), and schizophrenia [11], the brain mechanism associated with face recognition in SAD has not been well studied.

Some electrophysiological studies employing ERPs provide a source of evidence for specialized brain processes subserving face perception and recognition. In particular, N170 is described as a harmful component peaking at about 170 ms that is elicited by human faces [12, 13]. Because of the sensitive response to face stimulus, N170 is considered the specific component of face processing [14]. N170 as a classic face-specific component that reflects early-stage perception in the structural encoding of faces [15]. Since a study showed that N170 is not affected by the familiarity of the faces [16], it can be inferred that the familiarity processing is earlier than the early facial structural encoding process [17]. The N170 elicited by facial stimuli is mainly distributed on both sides of the posterior-temporal cortex. It mainly exhibits a larger amplitude on the right side of the posterior-temporal regions [18, 19]. It is proposed that N170 elicited by words would show a left-hemisphere dominance [20], while face stimuli elicited right-hemisphere dominance [21]. Except for upright faces, inverted faces have also been utilized as stimulus materials in face processing studies, which are supposed to destroy the configurational information related to face recognition [22]. In general, inverted faces delay the latency of N170, which is regarded as the main aspect of the N170 inversion effect [23, 24].

Some related studies showed that patients with SAD manifest many traits similar to other disorders, such as schizophrenia individuals, ASD patients, excessive Internet users (EIUs), and depressive patients [25]. In the early stage of face processing, characteristics of the N170 component revealed a lesion in EIUs or individuals with schizophrenia compared with normal individuals [11, 26]. The study also found that the abnormal early face processing of SAD patients was related to their response bias to unfamiliar faces. found that abnormality of early face processing in patients with SAD, which is associated with their response bias to stranger faces [6]. However, the associations between the aforementioned cognitive biases are unclear. Previous research on N170 in patients with SAD was mainly focused on the attentional bias of emotional expression but less on face recognition. Therefore, the primary purpose of this study was to explore the differences in face processing mechanisms between normal individuals and SAD patients before and after treatment by analyzing the N170 component. We also expected to find an indicator that could evaluate the improvement of patients' condition. We conducted a passive viewing upright and inverted emotional expression paradigm. We hypothesized to explore abnormality in latency or amplitude or the hemisphere effect of N170 in SAD.

## 2. Material and Methods

### 2.1. Participants

The study was carried out following the Declaration of Helsinki, and the experimental protocols used were approved by the institutional review board (IRB) of the Harbin Medical University. Twenty outpatients with SAD were recruited from the Psychology Department of Affiliated Hospital of Harbin Medical University, while 20 healthy control (HC) participants were recruited through advertisements. The patients with SAD were diagnosed using the validated Chinese translation of the Structured Clinical Interview for Diagnostic and Statistical Manual of Mental Disorders, Fourth Edition (DSM-IV) (SCID-IV), the gold standard for assessing SAD in China. Control participants were demographically matched HCs with no history of DSM-IV psychiatric disorders. These individuals were also screened using the SCID. All participants were right handed and reported no psychoactive substance abuse, no unstable medical illness, and no past or current neurological illness. The subjects' anxiety symptoms were assessed using the Brief Social Phobia Scale (BSPS) and the Interaction Anxiousness Scale (IAS). All participants provided written informed consent for the experiment. Participants with SAD and the matched HC were excluded because they dropped out of the therapy. We thus carried out the study using a sample of 12 patients with SAD and 12 HC participants. The groups did not differ in demographic characteristics. Compared to those in the HC-group, participants in the SAD group reported higher levels of social anxiety.

Twelve patients with SAD (5 men and 7 women) are between ages 19 and 24 years old (*M* = 21.50, SD = 1.51) who participated in the study. SAD patients were recruited by the Harbin Medical University (Daqing, China). For the healthy control (HC) groups, 12 subjects (7 men and 5 women) ranging in age from 18 to 25 years (*M* = 20.33, SD = 2.06) were recruited through a website. There were no gender, age, and educational level differences between patients with SAD and healthy control subjects. All subjects were screened by trained experts using the fourth edition version of the Diagnostic and Statistical Manual of Mental Disorders (DSM-IV) [27]. Patients with SAD were required to meet the criteria for social anxiety, while control subjects were required to confirm the absence of psychopathology. Exclusion criteria for both SAD and control subjects included bipolar disorder, schizophrenia, psychosis, delusional disorders, and an abnormal EEG. None of the SAD patients and healthy people reached the criteria for elimination.

Interaction Anxiousness Scale (IAS) [28] and the Brief Social Phobia Scale (BSPS) [29] were used to test the level of social anxiety. The total score of scales reflects the severity of the symptoms of SAD. A higher total score means a more severe condition. The prepatient group exhibited significantly higher scores (IAS: 58.00 ± 9.28, BSPS:42.33 ± 10.49) than HC-group (IAS: 30.58 ± 4.32, BSPS:7.25 ± 4.88), and the prepatient group exhibited significantly higher scores than the postpatient group (IAS: 43.83 ± 7.63, BSPS: 21.58 ± 12.39).

### 2.2. Stimulus Materials

The stimulus materials were a set of black-and-white schematic face pictures consisting of happy, neutral, and sad expressions. Each emotional expression included both upright and inverted faces. There were eighteen pictures for each condition (happy-upright, happy-inverted, neutral-upright, neutral-inverted, sad-upright, and sad-inverted) (see Figure 1). Such stimulating materials have already been used in research related to face recognition [30, 31]. Moreover, schematic faces demonstrate the main parts of a face enough to weaken gender differences in human faces.

### 2.3. EEG Recording

Electroencephalogram (EEG) signals were recorded from a 64-channel EEG amplifier (Synamps2 Compumedics Neuroscan) with a sampling rate of 1,000 Hz. Locations of electrodes followed the international 10–20 system. The impedance of all electrodes was kept below 5 KΩ. An electrode placed on the vertex served as the reference for online recording. The collected signals were re-referenced to the common average reference before further processing.

Notably, two datasets (before and one year after the treatment, respectively) of each patient with SAD were recorded under the same experimental conditions. The treatment was conducted by a clinical psychologist and a psychology teacher. Mainly, intensive intervention therapy was performed lasting 12 weeks. The form of intervention was a combination of group intervention and individual intervention. Patients were randomly assigned to an intervention group consisting of 6 people. The group of cognitive behavioral therapy was performed weekly, and the individual intervention was performed once a week, that is, each patient completed 12 group therapy sessions and 12 individual-therapy sessions. After one year, participants again completed an EEG recording and a scale evaluation.

### 2.4. Experimental Paradigm

Stimulus presentation was controlled by Eprime 2.0 (Psychology Software Tools, Inc.). Subjects were seated on a comfortable chair in front of the screen. All subjects were asked to reduce the body's movement during the experiment to minimize the impact of the electromyographic (EMG) artifacts. This study adopted the paradigm of passive viewing face pictures, which is most commonly used in face recognition [32, 33]. The detailed schematic diagram is illustrated in Figure 1(b). Each trial started with a training stage; meanwhile, pictures of six kinds of expressions were randomly presented for 300 ms. Subsequently, participants were instructed to press the button matching with the expression on a keyboard after sorting out the contents of the images. There was no time limit. The new round of the experiment would continue to start upon participants' responses. After the training phase, the subjects pressed the “SPACE” bar to start the formal experiment and formatted the same as the training phase. For the formal experiment, the picture of each case was randomly repeated four times and 68 times for each condition.

### 2.5. Data Analysis

The raw EEG data were filtered using the cut off frequency of 30 Hz Chebyshev low-pass filter (4-order IIR), which would weaken the powerline interference and EMG artifacts that are mainly above 30 Hz. Regardless, the remaining artifact-contaminated portions of the EEG were manually identified and excluded from further analysis.

Collected datasets consisted of patients before treatment (P-group-pre), one year after treatment (P-group-post), and healthy individuals (HC-group). The EEG was epoched offline from 50 ms before the beginning of the onset of the face to 500 ms after onset. In addition, epochs were averaged for every subject and for every class of stimuli. The baseline was corrected using 50 ms before stimulus onset. What's more, in this study N170 was identified as the most negative or negative ongoing peak between 106 and 192 from the grand-averaged waveform. To compare differences of emotional expression in similar subjects, repeated measures ANOVAs can examine specific effects or interactions.

The study of ERPs often used the asymmetry index (AI), to express asymmetry between the left and right brain hemispheres. AI is defined as *AI*=(*L* − *R*)/(*L*+*R*), where *L* and *R* are the values of the special regions of the left and right hemispheres [6, 34]. Previous research concluded that the response bias in individuals with SAD is resulted from impairments in early discrimination of social faces, as reflected by the absent early N170 differentiation effect, which was associated with their combined negative biases [6]. In this study, the N170-based asymmetry index (AI) was introduced to analyze the left- and right-hemisphere dominance of N170 for the three groups. For this experiment, since EEG mapping was obtained by using the normalized amplitude, AI was modified as follows:

(1) $$\begin{array}{c} AI_{N170-base\;d}=\frac{1}{N}\sum_{i=1}^{N}\left(X_{left}-X_{right}\right), \end{array}$$

where *N* is the number of the electrode and *X*_*left*_ and *X*_*right*_ are the normalized N170 amplitude of specific range in left and right hemispheres. Different value of *AI*_*N*170−*base*  *d*_ indicates the role that hemisphere dominance of N170 plays: (1) as the value is positive, it indicates that the N170 is dominant of right hemisphere; (2) as the value approaches zero, the left- and right-hemisphere dominance of N170 closes to balance; and (3) as the value is negative, it demonstrates that the N170 is dominant in the left hemisphere.

## 3. Results

### 3.1. N170 Topographical Distribution and Waveforms

EEG topographical mapping of N170 is displayed in Figure 2, and the value of each electrode was worked out by normalizing the average amplitude of a specific range. It could be seen that the right predominant N170 was mainly concentrated in posterior-temporal regions. Because of the topographical maps of N170, the electrodes of PO8 and PO7 (see Figure 2) as the most conspicuous sites were selected for further analysis. Moreover, Figures 3 and 4 depict the grand mean ERP waveforms under inverted or upright conditions, respectively. This graph shows that the main ERP components, including P1 and N170, were successfully induced and further proved the rationality of this experimental protocol.

### 3.2. N170 Amplitude

Irrespective of emotional expression, statistical tests were performed between groups according to upright and inverted conditions. The results revealed significantly enlarged N170 amplitude for P-group-pre relative to HC-group in inverted condition (*p*=0.02) and upright condition (*p*=0.02) at electrode PO8 but not at electrode PO7. A similar conclusion was also obtained for P-group-post versus HC-group. P-group-post showed greater N170 amplitude than HC-group in the right hemisphere both in inverted or upright stimuli (*p*=0.01 and *p*=0.004, respectively). Furthermore, analysis including the expression factors showed no significant amplitude difference in the left hemisphere and neither the right hemisphere.

### 3.3. N170 Latency for Different Groups

Table 1 depicts the mean and standard error of N170 amplitude and latency for inverted and upright conditions of PO7 and PO8. Across emotional expression, longer N170 latency was observed at PO8 under upright conditions for P-group-pre compared to P-group-post (*p*=0.002) and for H-group than P-group-post (*p*=0.002), but no significant difference was observed between P-group-pre and HC-group. Moreover, in hemisphere-independent analysis, except for P-group-pre, a longer N170 peak was elicited by inverted compared to upright faces within the other two groups (*p*=0.04 and *p*=0.03 for P-group-post and HC-groups).

### 3.4. AI Index Treatment Effect

In terms of N170 amplitude and latency, this study did not find the desired results reflecting the treatment effect. However, from P-group-pre to H-group the left-lateralized N170 was consistently enhanced after treatment in posterior-temporal regions as shown in Figure 2. Five symmetrical electrodes located in the posterior-temporal regions (PO7/PO8, PO5/PO6, P7/P8, P5/P6, and P3/P4) were taken one step further for examining hemisphere dominance, and formula (1) was then used for the next step. For this formula, *N* has a value of 5. The detailed values of *AI*_*N*170−*base*  *d*_ under inverted conditions or upright conditions are displayed in Table 2. According to Table 2, it could be clearly seen that from the first to the third column, the values of *AI*_*N*170−*base*  *d*_ exhibited a decreasing trend. When performing statistical analysis by using *t*-tests, significant differences were found in P-group-pre vs. P-group-post (*p*=0.04 (inverted) and *p*=0.04 (upright), respectively) and P-group-pre versus H-group (*p*=0.01 (inverted) and *p*=0.01 (upright), respectively) but not in P-group-post versus H-group.

### 3.5. Effects of Emotional Expression in SAD Patients

A three-factor ANOVA with repeated measures that can contact the significant differences between multiple emotional expressions was adopted. The factors were Hemisphere (2 levels: left, right), Orientation (2 levels: inverted, upright), and Emotional category (3 levels: happy, neutral, sad). The results showed that there were no significant main effects in latency (*F* (2.22) = 0.17, *p*=0.85) or amplitude (*F* (1.19, 13.04) = 0.09, *p*=0.81) of N170 in P-group-pre when comparing different emotional expressions. Furthermore, there was no any interaction with emotional expression.

## 4. Discussions

This study was conducted to study the differences in face processing mechanisms between patients with SAD before and after treatment and healthy people when looking at upright and inverted emotional expressions. The main results came from ERPs elicited by faces especially include a negative potential N170, which is considered to be the most persuasive component in face processing.

### 4.1. Processing Intensity of Early Face Recognition in SAD Patients

The two groups, group with SAD (P-group-pre) and HC-group, N170 amplitude, and latency were compared. It turned out that the P-group-pre of N170 amplitude was significantly larger than for the H-group? In the right hemisphere under upright and inverted conditions. The amplitude of N170 can reflect the processing intensity of early face recognition. Therefore, these data provide evidence that a greater processing intensity of SAD patients in the right hemisphere was responsible for the abnormalities during the process of early face recognition. In this regard, this study did not investigate the differences between P-group-post and H-group. The main reason was to get rid of a certain degree of “expert effect” produced by previous experiments on the impact of N170 amplitude [18].

### 4.2. Inversion Effect in SAD Patients

For face recognition, the research on the inversion effect has always been a popular topic for decades. Face inversion delays and/or enhances the N170 component [26]. Furthermore, previous literature has shown that gestalt-based schematic faces that lack physiognomic components may inhibit a holistic perception of a face and do not trigger the analysis of the components when the face is inverted [35]. Due to this study's usage of schematic faces as stimulus materials, it is understandable that the inversion effect did not manifest itself in the facets of amplitude. In this study, the inversion effect, therefore, showed up as a delay of N170. It is well known that an inverted image disrupts the configurational information of face recognition. The accepted result is that the latency of N170 in healthy people will have a noticeable difference in upright faces related to inverted faces [36, 37]. Irrespective of hemisphere, for both the P-group-post and H-group, the intragroup statistic test exhibited a significant difference when comparing N170 latency in upright faces with inverted faces, while P-group-pre did not reveal any differences in this respect. Therefore, it can be inferred that there was no inversion effect in SAD patients. Given that the autism inversion effect was not observed before, this study assumes that patients with SAD may have the same face processing strategies as those with autism. Feature-based processing methods different from the healthy people were adopted for individuals with ASD [38, 39].

### 4.3. Whether the Emotional Expression Can Modulate N170 in SAD Patients

The ANOVA was used to explore the effect of emotional expression in SAD patients for P-group-pre in follow-up studies. The results revealed that there is no significant difference associated with the factor of emotion. Whether it can enhance the processing of emotional expression in patients has been controversial. Numerous studies hold that SAD could lead to a general overactivation of the brain when processing any emotional faces [39]. On the contrary, other studies have demonstrated that SAD and emotional expression are irrelevant. Studies have proved that scary faces (typical: angry) can induce specific responses in patients with SAD [40]. The sad expression conveyed avoidance or seeking for protection without directly displaying hostility in the patients with SAD. The above may be one of the reasons why SAD patients are not sensitive to emotion in this study. In short, under the same experimental protocol and stimulus materials, schematic faces of different emotional expressions cannot modulate N170 in SAD patients.

### 4.4. The Change in Hemisphere Dominance during the Treatment

Regarding the distribution of the central brain regions of N170 elicited by face-related materials, the general conclusion is that posterior-temporal regions on both sides, especially the right hemisphere, can induce the maximum amplitude of N170. However, in this study, mainly a left-lateralized N170 was observed in H-group. A similar phenomenon was reported in some research studies adopting text-related stimuli [20]. In this regard, this study provided two reasonable explanations. First of all, colorless and explicit stimulus materials did not activate the right hemisphere, which is responsible for painting, geometry, and other functions [41, 42]. Another line-shaped stimulating material used in this study may be identified as Chinese characters. For example, a round face is like a “口” word, and the eyes, nose, and mouth together make up “土” or “工” word. On the contrary, a right-lateralized N170 was found in P-group-pre. Unlike ordinary people, some studies reported that for patients with SAD, the suitable posterior-temporal regions or right amygdala could be activated by emotional or line-shaped faces (such as schematic faces) [10, 28, 43]. Based on the findings in this study, we first put forward that under inverted conditions or upright conditions, the change in the value of *AI*_*N*170−*base*  *d*_ can be used as an indicator of condition improvement in SAD patients.

## 5. Conclusions

To sum up, according to a protocol of face recognition, this study adds new value that under inverted conditions or upright conditions the change in the value of *AI*_*N*170−*base*  *d*_ can be used as an electrophysiological indicator of treatment improvement in patients with SAD. Besides, this study reveals no inversion effect in patients with SAD, suggesting that abnormal facial perception in patients with SAD may be similar to other patients with dysfunctional social ability, e.g., autism.

There are several limitations in this study. First, the behavioral data of reaction time were not recorded. The experiment does not mark when subjects press the button, so the reaction time of different expressions cannot be calculated. Second, while this study puts forward that similarities in a face processing stage may exist between patients with SAD and with ASD, no further experiment was designed to address it. It requires future research to understand it. However, the AI approach is a way to illustrate our conclusion, and the next step is to explore the difference between AI and other approaches. Third, the main limitation is the small sample size. It requires more participants and future research to verify the conclusion.

## Figures and Tables

**Figure 1:** The stimulus materials of the experiment (a) and a schematic representation of the experimental protocol (b).

**Figure 2:** (a) The grand-averaged N170 amplitude mapping under inverted conditions and (b) upright conditions. The topographic map on the left was the prepatient group, and the middle and right for the postpatient group and the HP-group, respectively.

**Figure 3:** Grand mean ERPs in response to happy, neutral, and sad faces for (a) prepatient group, (b) postpatient group, and (c) HP-group at electrodes PO7 (left) and PO8 (right). The ERP was elicited by inverted stimuli.

**Figure 4:** Grand mean ERPs in response to happy, neutral, and sad faces for (a) prepatient group, (b) postpatient group, and (c) HP-group at electrodes PO7 (left) and PO8 (right). The ERP was elicited by upright stimuli.

**Table 1:** Means (and standard deviations) for latency and amplitude of N170.

Electrode	Condition	Latency (ms)	Amplitude (*u*V)
Prepatient group			
PO8	Inverted faces	158.97 (13.34)	−3.17 (2.20)
	Upright faces	154.47 (16.75)	−3.12 (2.10)
PO7	Inverted faces	154.58 (18.98)	−2.93 (1.79)
	Upright faces	149.03 (18.38)	−3.07 (1.99)

Postpatient group			
PO8	Inverted faces	153.58 (18.86)	−3.13 (1.74)
	Upright faces	144.83 (18.62)	−3.34 (1.99)
PO7	Inverted faces	147.75 (24.76)	−3.03 (1.67)
	Upright faces	142.14 (22.87)	−3.18 (1.50)

HC-group			
PO8	Inverted faces	158.94 (14.00)	−2.23 (1.15)
	Upright faces	153.92 (15.21)	−2.21 (1.20)
PO7	Inverted faces	160.00 (13.21)	−3.19 (2.05)
	Upright faces	155.17 (14.59)	−3.30 (2.21)

**Table 2:** The values (and standard deviations) of *AI*_*N*170−*base*  *d*_ in three groups under inverted and upright conditions.

	Prepatient group	Postpatient group	HC-group
Inverted faces	0.1565 (0.39)	0.0115 (0.41)	−0.0341 (0.42)
Upright faces	0.1420 (0.37)	−0.0074 (0.43)	−0.0412 (0.45)

## Data Availability

The data used to support the findings of this study are available from the author upon request.
